The article "Mannosylated Chitosan Nanoparticles for Delivery of Antisense Oligonucleotides for Macrophage Targeting" was retracted in 2021. Reasons: manipulated images; duplicated images; original data or images not available; concerns about the data.

# Mannosylated Chitosan Nanoparticles for Delivery of Antisense Oligonucleotides for Macrophage Targeting

**DOI:** 10.1155/2014/526391

**Published:** 2014-06-26

**Authors:** Gyati Shilakari Asthana, Abhay Asthana, Dharm Veer Kohli, Suresh Prasad Vyas

**Affiliations:** ^1^Maharishi Markandeshwar College of Pharmacy, Maharishi Markandeshwar University, Mullana Ambala, Haryana 133207, India; ^2^Department of Pharmaceutical Sciences, Dr. Hari Singh Gour Vishwa Vidyala, Sagar, Madhya Pradesh 470003, India

## Abstract

The therapeutic potential of antisense oligonucleotides (ASODN) is primarily dependent upon its safe and efficient delivery to specific cells overcoming degradation and maximizing cellular uptake *in vivo*. The present study focuses on designing mannosylated low molecular weight (LMW) chitosan nanoconstructs for safe ODNs delivery by macrophage targeting. Mannose groups were coupled with LMW chitosan and characterized spectroscopically. Mannosylated chitosan ODN nanoparticles (MCHODN NPs) were formulated by self-assembled method using various *N*/*P* ratio (moles of amine groups of MCH to phosphate moieties of ODNs) and characterized for gel retardation assay, physicochemical characteristics, cytotoxicity and transfection efficiency, and antisense assay. Complete complexation of MCH/ODN was achieved at charge ratio of 1:1 and above. On increasing the *N*/*P* ratio of MCH/ODN, particle size of the NPs decreased whereas zeta potential (ZV) increased. MCHODN NPs displayed much higher transfection efficiency into Raw 264.7 cells (bears mannose receptors) than Hela cells and no significant toxicity was observed at all MCH concentrations. Antisense assay revealed that reduction in lipopolysaccharide (LPS) induced serum TNF-*α* is due to antisense activity of TJU-2755 ODN (sequence complementary to 3′-UTR of TNF-*α*). These results suggest that MCHODN NPs are acceptable choice to improve transfection efficiency *in vitro* and *in vivo*.

## 1. Introduction

Gene therapy is a potential approach to cure or prevent diseases through gene expression before the transcription stage [1]. It includes approaches based on utilization of deoxyribonucleic acid (DNAs), oligodeoxyribonucleotides (ODNs), small interference RNAs (SiRNA), and so forth for treatment and mitigation of diseases. Oligonucleotides based therapeutic techniques have attracted much attention because they provide a rational way to design antisense oligonucleotides (As-ODN), decoy oligonucleotides that bind to DNA-binding regulatory proteins, and siRNA/miRNA that suppress specific gene expressions. ODNs with base sequences complementary to a specific RNA have offered the exciting potential to selectively modulate the expression of an individual gene and, thus, possess the potential for activity in the treatment of viral infections or cancer. ODNs include a new generation of antiviral, antitumoral, and anti-inflammatory agents, in various categories [2–4]. As-ODNs are anionic, large molecular weight (5–10 kDa), 10–30 nucleotide bases sequence of short single strands of DNA; RNA their analogs molecules designed to modulate gene expression [5] and possessing high hydrophilicity [6]. For antisense applications, ODNs interact and form a duplex with their complementary target mRNAs or pre-mRNAs through Watson-Crick base pairing in a sequence-specific manner and then inhibit their translation [7, 8]. Therefore the genetic code in the RNA cannot be read, which consequently inhibits production of the disease-causing protein [1]. At the molecular level, several mechanisms of antisense actions have been proposed for antisense drugs. These include inhibition of transcription, inhibition of splicing, and inhibition of mRNA maturation [9]. Among them, activation of RNase H is by far one of the most recognized theories accepted by many researchers. After entering cells, ODNs hybridize to the target mRNA and form a sense-antisense RNA DNA duplex. For therapeutic application, antisense technology promises greater advantages over drugs currently on the market by offering new types of drugs that are easy to design and have a very high molecular target selectivity and efficacy, inhibiting a specific gene expression, and an expected low toxicity due to metabolism to natural nucleotide components by the endogenous systems [5, 10]. Vitravene, is only ODN based therapeutic (antisense ODN) approved by FDA and several others are in Phase 3 clinical trials. However, ODNs therapeutics have been associated with multiple obstacles, that is, poor physiological stability and cellular uptake [11, 12], inadequate intracellular ODNs concentration [13, 14], inability to target specific cell [14, 15], lack of tissue specificity [16], and nuclease degradation [14, 17]. Thus, intracellular delivery and therapeutic applications in diseases of ODN-based therapeutics have been compromised. Although various chemical modifications of ODNs can be used to overcome these problems [18], they offer other limitations such as low binding affinity, nonsequences specific biological effects, toxicity, and acute homeostatic changes after* in vivo* administration [19–23]. Therefore, development of effective delivery systems that are capable of protecting and efficiently deliver ODNs intracellularly in target cells becomes essential to exploit the promising applications offered by successful ODN delivery. Among the gene delivery vectors, nonviral vectors are preferred due to its ease of synthesis, low immunogenicity, and unrestricted gene materials size in addition to potential benefits in terms of safety [24–27].

The article "Mannosylated Chitosan Nanoparticles for Delivery of Antisense Oligonucleotides for Macrophage Targeting" was retracted in 2021. Reasons: manipulated images; duplicated images; original data or images not available; concerns about the data.

Nanoparticles (NPs) were introduced as nonviral gene vectors to solve issues related to ODNs delivery [28–36]. Other carriers such as microspheres, matrices, complexes with polycations, and starburst dendrimers have been recently investigated [10, 37–40]. The major advantage of using nanocarriers resides in the possibility of conjugating ligands to them as to direct them to a desired site for localized delivery in cells, tissue, or organ [41]. ODNs in complex state with nanocarriers avail protection against nuclease degradation [38, 42–44]. Further, their cell uptake could be increased as carrier-ODNs complexes are taken up through active endocytosis process.

Recently, biodegradable nanoparticles have been studied as potential inert and biocompatible carriers for genetic materials, for example, polylactide polyethylene glycol (PLA-PEG), cationic polystyrene spongelike alginate, polyalkylcyanoacrylate, poly isohexylcyanoacrylate or poly isobutylcyanoacrylate, and albumin chitosan nanoparticles [36, 45–51].

Among the large number of cationic polymers described, chitosan is shown to be an effective vector because of condensing and delivered DNA, siRNA* in vitro* and* in vivo* [52, 53], and ODN* in vitro* [54]. It is a natural positively charged polymer that can be utilized for preparation ofnanoparticulate carriers which represents a novel strategy for the safe and efficient delivery of gene. It has been extensively examined for its potential in the development of controlled release drug delivery formulation due to its unique polymeric cationic characteristic gel forming and film forming properties [55, 56]. Chitosan has beneficial qualities such as low toxicity, low immunogenicity, excellent biodegradability, and biocompatibility [57, 58]. It is a suitable candidate for gene delivery system due to its ability to spontaneously form interpolyelectrolyte stable complexes with genetic material (ODNs or DNA) as a result of cooperative electrostatic interactions between the positive amino groups of chitosan and the negative phosphate groups of DNA/ODN [54, 56, 59].

Consequently, several groups have conducted studies using chitosan/DNA nanoparticles, including use of galactosylated chitosan [60], galactosylated chitosan-graft-poly(vinylpyrrolidone) (PVP) [61], mannosylated chitosan/DNA nanoparticles [62], trimethylated chitosan oligomers [63], N-dodecylated chitosan [64], deoxycholic acid modified chitosan [65], galactosylated chitosan/ODN vector [54], or ligand attached chitosans for targeting cell membrane receptors [66]. However, chitosan was difficult to solubilize in water and was dissolved in acidic solution. Low molecular weight water soluble chitosan has been employed, which is highly water soluble and forms complex with plasmid DNA/ODN at physiological pH [54, 67, 68]. They can display high transfection efficiency along with the higher plasmid DNA/ODN loading, protection against the nuclease degradation, and being less toxic [54, 69, 70]. Ligands are molecular extension that pave fate of delivery system for active targeting and increase overall therapeutic potential. Thus the receptor mediated gene targeting is a promising approach to obtain cell-selective gene transfection. A number of receptor mediated gene delivery systems have been developed to introduce the foreign DNA/ODN into specific cell types. Ligands currently being investigated include galactose [71–80], mannose [66, 81–85], lactose [86], transferrin [87, 88], and epidermal growth factor [89]. Active targeting using receptor mediated interaction has been effective in gene delivery [90].

The article "Mannosylated Chitosan Nanoparticles for Delivery of Antisense Oligonucleotides for Macrophage Targeting" was retracted in 2021. Reasons: manipulated images; duplicated images; original data or images not available; concerns about the data.

Among the various receptors, asialoglycoprotein receptors and mannose receptors are the most promising for gene targeting because they exhibit high affinity and are rapidly internalized [91]. Wide variety of macrophages (including Kupffer cells) express mannose specific membrane receptors, which internalize glycoprotein bearing mannose residue via clathrin-coated vesicles, to allow a delivery into the endosomal system [91–94].

In gene delivery systems, the mannosylation of cationic polymers, such as mannosylated polylysine and PEI, were used to achieve the delivery of gene to macrophages [82, 85]. Mannosylated chitosan for plasmid DNA has also been reported earlier for macrophage targeting [95].

Although chitosan has been studies for more than a decade as a gene vector for DNA, ODN, and siRNA [54, 96], so for to our knowledge, there is no study that has been carried out to investigate the use of mannosylated chitosan nanoparticles to determine ODN* in vitro*. In the present study, we formulate mannosylated LMW-water soluble chitosan formulations by self-assembled method, characterized for gel retardation assay, particle size, particles shape, and particles surface morphology and zeta potential, complexing capacity, protection ability, and MCHODN NPs stability. Cytotoxicity studies, transfection efficiency, and antisense assay were also assessed for developed nanoparticles formulations.

## 2. Materials and Methods

The phosphorothioate modified AS ODN used in this study, TJU-2755, designed to target the 3′-UTR of the primary RNA transcript of TNF-*α*, was synthesized by Sigma Aldrich. The sequence of TJU-2755 is 5′-TGATCCACTCCCCCCTCCACT-3′; random sequence of ODN is 5′-CCTCCACTGCTACCTCACCTC-3′; FITC-ODN was also received from Sigma Aldrich. Water-soluble LMWC with a molecular weight of 22 KDa, with degree of deacetylation of 72.5%, was received from Kittolife Co., Seoul, Republic of Korea. Oligreen reagent was purchased from Molecular Probs Inc. (Netherlands); RAYBio@ rat TNF-alpha ELISA kit was purchased from RAYBio Ltd. Mannopyranosyl phenyl isothiocyanate, dimethyl sulfoxide (DMSO), and Tris Borate EDTA were purchased from Sigma Aldrich. All other chemicals were obtained commercially as reagent grade products.

The article "Mannosylated Chitosan Nanoparticles for Delivery of Antisense Oligonucleotides for Macrophage Targeting" was retracted in 2021. Reasons: manipulated images; duplicated images; original data or images not available; concerns about the data.

## 3. Preparation of Mannosylated Chitosan (MCH)

Mannosylated chitosan (MCH) was prepared by previously reported method with slight modifications [61]. Briefly, 120 mg of accurately weighed water-soluble LMWC was dissolved in 2 mL of double distilled water (2 mL) and mixed with solution of mannopyranosyl phenyl isothiocyanate (Sigma Co. St. Louis, India) in 1 mL of DMSO. The solution was stirred for 24 h at room temperature (24°C). The MCH was precipitated by adding 10 volumes of isopropanol and centrifuged at 13,000 rpm for 15 min. After repeating this process five times, the pellets were dried in vacuum oven. The MCH composition was determined by FT-IR and proton nuclear magnetic resonance spectroscopy (1H NMR, 600 MHz; Bruker, Germany). The degree of sugar substitution was determined by the sulfuric acid micromethod [97].

## 4. Preparation of MCHODN Nanoparticles (MCHODN NPs)

MCHODN nanoparticles were prepared by self-assembling methods as reported earlier with slight modifications [62]. MCHODN charge ratio (*N*/*P*) was expressed as the ratio of moles of the amine groups of MCH to those of the phosphate moieties of ODNs. Nanoparticles were induced to self-assemble in phosphate buffer (pH 7.4) by mixing ODN with required polymer solution at the desired ratio. The complexes were allowed to stand at room temperature for 1 h. The complex formation was confirmed by gel retardation assay with 1% agarose gel.

## 5. Characterization of MCHODN Nanoparticles

### 5.1. Gel Retardation Assay

The formation of MCHODN NPs was determined by using gel retardation assay. Agarose gel was prepared with 1% agarose solution in Tris-borate-EDTA (TBE: 4.45 mM Tris base, 1 mM sodium EDTA, 4.45 mM boric acid pH 8.3) buffer. A series of different *N*/*P* ratio of MCHODN nanoparticles were loaded in the well (20 *μ*L of the sample equivalent to 0.2 *μ*g of ODN). A 1 : 6 dilution of loading dye was added to each well and electrophoresis was carried out at a constant voltage of 55 V for 2 h in Tris Borate EDTA (TBE) running buffer containing 0.5 *μ*g/mL ethidium bromide. The bands of ODN were then visualized under a UV illuminator.

The article "Mannosylated Chitosan Nanoparticles for Delivery of Antisense Oligonucleotides for Macrophage Targeting" was retracted in 2021. Reasons: manipulated images; duplicated images; original data or images not available; concerns about the data.

### 5.2. Measurement of Particle Size and Zeta Potential

Size of the nanoparticles was determined in triplicates by photon correlation spectroscopy (PLS) using Zetasizer, Nano ZS (Malvern Instruments Ltd., Malvern, Worcestershire, UK). The particle size analysis of the nanoparticles was performed at 25°C, an angle of 90° for the photomultiplier, and a wavelength of 633 nm. The surface charge (zeta potential) of the nanoparticles was determined from the electrophoretic mobility. The zeta potential measurements were performed at pH 7.4 in triplicates using the 100 *μ*L aqueous dip cell by Zetasizer, Nano ZS (Malvern Instruments Ltd., Malvern, Worcestershire, UK). The samples were diluted 1 : 100 with double distilled water before measuring.

### 5.3. Shape and Surface Morphology

#### 5.3.1. Transmission Electron Microscopy (TEM)

Morphological examination of MCHODN nanoparticles at *N*/*P* ratio 3 : 1 was investigated by transmission electron microscopy** (**TEM, JEM 1200, EX 11, JEOL, Japan). One drop of sample was placed on a copper grid and negatively stained with uranyl acetate (1% w/v) solution for 30 s. The grid was allowed to dry further for 10 min and examined under the transmission electron microscope [98, 99].

#### 5.3.2. Scanning Electron Microscopy (SEM)

A drop of the MCHODN nanoparticles preparation was dried on a polished aluminium surface and the sample was sputtered with gold for 30 s under argon atmosphere (Agar sputter coater). Thereafter SEM was performed with S-4500 Hitachi field emission electron microscope (Krefeld, Germany) with the upper detector at 25 KV [100].

### 5.4. Determination of ODN Association Efficiency

ODN association efficiency of the MCHODN NPs was evaluated using the method as reported by Huang et al. [99] with slight modification. To measure the association efficiency of ODN, 16 *μ*L of the MCHODN NPs was spun down at 15,000 rpm for 30 min (Avanti J-25 centrifuge, Beckman Coulter Inc., Fullerton, CA, USA). The supernatant was mixed with 1 mL working OliGreen reagent and ODN content was estimated spectrofluorimetrically at 480 nm and a 520 nm excitation and emission, respectively [101, 102]. ODN association efficiency (%) of NPs is the amount of condensed ODN (difference between the total amount of ODN used for the NPs preparation and the amount of nonentrapped ODN remaining in the supernatant) calculated as a percent of the total amount of ODN used.

### 5.5. Resistance of MCHNP/ODN against DNase I Digestion and Release Assay

Protection and release assay of ODN in nanoparticles were carried out by gel electrophoresis, following the reported procedure [103]. To assess the stability against nuclease digestion, free ODN and MCHODN nanoparticles (0.2 *μ*g) with various *N*/*P* ratios were separately incubated with DNase I (10 U) in DNase digestion buffer containing 50 mM, Tris-Cl, pH 7.6, and 10 mM MgCl_2,_ at 37°C for 1 h. After DNase I digestion, all the samples were treated with 4 *μ*L of 25 mM EDTA for 10 min to inactivate the DNase I and mixed with 20 *μ*L sodium dodecyl sulfate (SDS, 1.0% by dissolving in 0.1 N NaOH, pH 7.2)). To dissociate the ODN from MCH, the reaction mixtures were incubated in BOD incubator at 60°C overnight. After phenol/chloroform extraction, the ODN was precipitated with cold isopropanol. The pellets were dissolved in 10 mL of TBE buffer and applied to a 1.0% agarose gel electrophoresis for 40 min at 100 V [103].

The article "Mannosylated Chitosan Nanoparticles for Delivery of Antisense Oligonucleotides for Macrophage Targeting" was retracted in 2021. Reasons: manipulated images; duplicated images; original data or images not available; concerns about the data.

### 5.6. Stability of MCHODN NPs

#### 5.6.1. Dispersive Stability of Nanoparticles

The procedure reported by Kim et al. [103] with slight modifications was followed to estimate dispersing stability of NPs. Briefly, the nanoparticles formulations were dispersed in 10 mM phosphate buffer containing 150 mM NaCl and the dispersive stability of nanoparticles was evaluated by turbidity measurement spectrophotometrically at 340 nm. The results are given in Figure 7. Also serum stability of** e**ach of the formulations was observed in the presence of fetal bovine serum (18 *μ*L DMEM medium was taken with 2 *μ*L of FBS). The samples were incubated at 37°C with mild agitation and evaluated by agarose gel electrophoresis at 0.25, 0.5, 1, 1.5, and 2 days. The results are shown in Figure 8.

### 5.7. *In Vitro* Cell Line Study

#### 5.7.1. Cell Lines and Cell Culture

Raw 264.7 (murine macrophage cell line expressing moderate mannose receptors) [62] and Hela (human cervix epithelial g cells) cells were procured from the NCCS Pune (MHA India). Both cell lines were maintained in Dulbecco's modified Eagle medium (DMEM, Sigma, India) supplemented with 10% fetal bovine serum (FBS), streptomycin (100 *μ*g/mL), and penicillin (100 U/mL). The cells were incubated at 37°C in a humidified atmosphere containing 5% CO_2_/95% relative humidity (CO_2_ Incubator; Binder, Germany). Trypsin/EDTA medium was used to split the cells.

#### 5.7.2. Cell Viability Study

*In vitro* cytotoxicity assay was performed as per reported method [54] to evaluate the effect ofpolymer (mannosylated chitosan) concentration and oligonucleotide concentration on cell viability of Raw 264.7 cells and Hela cells. The cell growth inhibition activity of samples was evaluated by 3-(4,5-dimethylthiazol-2yl)-2,5-diphenyl tetrazolium bromide (MTT) colorimetric assay. Briefly, both cell lines were maintained in Dulbecco's modified Eagle medium (DMEM) under suitable conditions as mentioned above. When the cells were confluent, they were seeded into 96-well culture plates at a cell density of 1 × 10^4^ cells/well and the plates were maintained under the conditions previously mentioned for twenty-four hours. Therefore, the old medium was carefully aspirated and the cells were incubated in 100 *μ*L serum free medium with various amounts of polymer (concentrations ranging from 5 to 200 *μ*g/mL of and man-chitosan).

The article "Mannosylated Chitosan Nanoparticles for Delivery of Antisense Oligonucleotides for Macrophage Targeting" was retracted in 2021. Reasons: manipulated images; duplicated images; original data or images not available; concerns about the data.

After 16 h, the medium was removed and the cells were rinsed twice with 1x PBS. The wells were refilled with complete medium and cells were cultured for another 24 h. 10 *μ*L of MTT dye solution (5 mg/mL) was added into each well and the plate was incubated for 4 h at 37°C allowing viable cells to reduce the MTT into purple colored formazan crystal [104]. The medium was later removed and 150 *μ*L of dimethylsulfoxide (DMSO) was added to each well and the plate was incubated for 30 min at room temperature. The optical density was measured at 550 nm. DMSO was used to dissolve the formazan crystals.

The cell viability was expressed as percentage compared to a control that had not been treated with polymers, using the following equation:

(1) $$\begin{array}{c} \text{Cell}\;\text{Viability}\;\left(\%\right)=\left(\frac{N_{i}}{N_{c}}\right)\times 100\;\text{or}\\ \text{Cell}\;\text{Viability}\;\left(\%\right)=\left(\frac{{\text{OD}}_{590}\;\text{sample}}{{\text{OD}}_{590}\;\text{control}}\right)\times 100, \end{array}$$

where *N*_*i*_ and *N*_*c*_ are the number of surviving cells in the group treated with ODN associated formulation and in the untreated cell group, respectively, or where the OD_590_ sample represents the measurement from the wells treated with polymer and OD_590_ control represents the wells treated with PBS buffer only.

In order to investigate the effect of ODN concentration on cell viability, another set of experiments was performed in the same manner as above. After 24 h of incubation of cells (1 × 10^4^ cells/well), 100 *μ*L serum free medium containing different amount of ODN (1, 5 and 10 *μ*g) either free or in MCHODN NPs was added into each well and cells were incubated for same period of time under the conditions mentioned earlier and cell viability was also determined.

#### 5.7.3. Transfection with Complexes* In Vitro*

In a transfection assay, Raw 264.7 cells and Hela cells were seeded at the density of 5.0 × 10^5^ cells/dish in 60 mm culture dishes with 5 mL of complete medium (Dulbecco's modified Eagle containing 10% serum DMEM) and incubated for 24 h prior to transfection. Transfection was performed on cells that were approximately 70% confluent. Before transfection, the complete medium was removed and cells were rinsed once with 1x PBS. The naked ODN and MCHODN NPs (containing 10 *μ*g of ODN) were diluted in 2 mL DMEM medium and then were used to refill the dishes, and incubated at 37°C for 6 h. Thereafter, serum and DMEM medium were added to these dishes to make up the final volume of medium to 5 mL containing 10% serum. Transfection with Lipofectin (GIBCO BRL) was carried out as positive control according to manufacturer's protocol. After another 18 h, the medium containing nanoparticles was removed. The cells were rinsed twice with 1x PBS, harvested, and resuspended in 1x PBS. ODN concentration in cell lysate was determined spectrofluorimetrically at excitation and emission wavelengths of 495 nm and 520 nm, respectively.

The article "Mannosylated Chitosan Nanoparticles for Delivery of Antisense Oligonucleotides for Macrophage Targeting" was retracted in 2021. Reasons: manipulated images; duplicated images; original data or images not available; concerns about the data.

#### 5.7.4. Competition Assay

Competition assay was carried out to confirm the uptake of MCHODN nanoparticles mediated by mannose receptor by adding different amount of mannose (10, 20, and 50 mM of the final volume) as a competitor for mannose in MCHODN NPS. Raw 264.7 cells were preincubated for 15 min with different amount of mannose, and transfection assays by using MCH/ODN NPs prepared at charge ratio 3 : 1 were conducted as described previously. All experiments were performed in triplicate [62].

### 5.8. Quantification of ODNs in Cells

ODN concentrations in cell lysate were determined spectrofluorimetrically as reported earlier [105–107]. After incubation period, transfection medium was removed and cells were washed three times with ice cold PBS (8 g/L NaCl, 0.2 g/L KCl, 1.56 g/L Na_2_HPO_4,_ and 0.2 g/L KH_2_PO_4_ in water at pH 7.2). The cell lysate was obtained after cells lysis with 0.2 mL of 1% Triton X-100 in 50 mM Tris-HCl buffer (pH 8.0). The cell lysate solutions were determined by LB05 spectrofluorophotometer (Shimadzu, Japan, *λ*ex, 492 nm *λ*em 519 nm) to quantify cell associated FITC ODN concentrations. The unknown concentration of ODN was determined by extrapolation from standard curve. Transfection efficiency is expressed as the amount (ng) of ODN per well of cells.

### 5.9. Cell Uptake Study

#### 5.9.1. Fluorescence Microscopy

Cellular accumulation of FITC-SODN was examined using fluorescence microscopy as reported earlier [108]. In these studies, Raw 264.7 cells were plated on 24-well plates at a density of 5 × 10^5^ cells/well in 3 mL complete medium (DMEM containing 5% FBS) and incubated for 24 h. The complete medium was removed and cells were rinsed once with 1x PBS. Then cells were incubated with free FITC-ODN or FITC-MCHODN NPs at 3 : 1 MCH/ODN ratio for 4 h at 37°C, washed three times with ice-cold PBS, and fixed with 4% (v/v) paraformaldehyde inPBS for 15 min at room temperature and again washed four times with PBS. The cells were analyzed by fluorescent microscope (Nikon, Japan).

The article "Mannosylated Chitosan Nanoparticles for Delivery of Antisense Oligonucleotides for Macrophage Targeting" was retracted in 2021. Reasons: manipulated images; duplicated images; original data or images not available; concerns about the data.

#### 5.9.2. Confocal Laser Scanning Microscopy (CLSM)

Raw 264.7 cells were plated on six-well microplates at a density of 5 × 10^5^ cells/well and incubated with free FITC-ODN or FITC-ODNnanoparticles at 3 : 1 MCH/ODN ratio for 4 h at 37°C, washed three times with ice-cold PBS, fixed with 4% (v/v) paraformaldehyde in PBS for 15 min at room temperature, and again washed four times with PBS. For staining nuclei, fixed cells were permeabilized with 0.2% Triton X-100-PBS for 20 min, stained with DAPI, washed once with 1 mL of cold PBS, and mounted on slide glasses with 50% glycerol-2.5% DABCO (1,4-diazabicyclo-[2,2,2] octane) (Sigma Chemical Co., Inc., St. Louis, MO)-PBS. Then the fluorescence images were acquired with a Zeiss 510 Meta confocal microscope.

### 5.10. Antisense Efficacy of ODN Delivered by Nanoparticulate Formulations (MCHODN NP2 and Free ODN Solution)

The* in vitro* suppressive effect of ODN in Raw 264.7 cells was determined using a method reported earlier with slight modifications [62, 109]. Raw 264.7 cells were seeded at a density of 3 × 10^5^ cells in a 24-well plate and cultured for 18 h, transfected with MCHODN NPs and free ODN solution by addition into a 24-well plate, and incubated for 6 h. To this serum and serum-free growth medium (DMEM) was added and incubated for another 18 hours at 37°C. After 24 h the cells were challenged with 100 ng/mL lipopolysaccharide (LPS). Two hours later, the culture medium was removed and stored at −70°C. The content of TNF-*α* in cell culture supernatant was evaluated using ELISA.

## 6. Results and Discussion

Despite its superiority as a biomaterial, chitosan is not fully soluble in water; however, it is readily soluble in acidic solution. Aqueous solubility of chitosan only in acidic solution limits its application to bioactive agents such as gene delivery carriers, peptide carriers, and drug carriers.

Water-soluble chitosan is easily soluble in aqueous solution with neutral pH. Its advantages are ease of modification useful as gene/peptide drug carriers and drug carriers [67, 110, 111].

### 6.1. Spectroscopic Analysis

Chitosan exhibits the characteristic bands of –NH_2_ scissoring vibrations at 1657 cm^−1^, carbonyl asymmetric stretching vibrations at 1564 cm^−1^, and C–O stretching vibrations of the pyranose ring at 1071 cm^−1^ (Figure 1). NMR spectrum of chitosan is shown in Figure 2. The solvent used was D_2_O and *δ* value from 1H NMR at 3.2 to 3.1 shows characteristic peaks of –CH_3_– second carbon of chitosan.

The article "Mannosylated Chitosan Nanoparticles for Delivery of Antisense Oligonucleotides for Macrophage Targeting" was retracted in 2021. Reasons: manipulated images; duplicated images; original data or images not available; concerns about the data.

Mannosylated chitosan (MCH) was synthesized by the reaction between amine groups of chitosan and isothiocyanate groups of *α*-D-mannopyranosyl phenyl isothiocyanate as shown in Scheme 1. The composition of MCH was determined by FTIR (Figure 3) and 1H NMR (Figure 4). The MCH exhibited the characteristic band of mannose at 808 cm^1^ and 890 cm^−1^, COO asymmetric stretching vibration at 1626 cm^−1^, and COO symmetric stretching at 1417 cm^−1^ and characteristic *δ* value from 1H NMR at 7.1 (–CH– of mannopyranosyl phenyl isothicyanate) and 2.1 (–CH_3_ of chitosan) (Figure 4). The substitution value of mannose coupled with water soluble chitosan was 5.9 mol %.

## 7. Characterization of MCHODN Nanoparticles

### 7.1. Gel Retardation Assay of MCHODN Nanoparticles

The positive charge of mannosylated chitosan and negative charge on ODN have tendency to enforce electrostatic interactions between them to form MCHODN nanoparticles. The confirmation of nanoparticles formation between MCH and ODN was evaluated by gel retardation assay. The nanoparticles were analyzed in 1.0% agarose gel electrophoresis Figure 5.

It shows the influence of charge ratios on ODN condensation by MCH from gel retardation assay. The results indicate that migration of ODN in gel was retarded with increasing the proportion of MCH to ODN. In present assay the *N*/*P* ratio of MCH to ODN was determined at which a given amount of ODN is completely complexed by MCH. This ratio was visualized by the gel retardation assay after subsequent staining with ethidium bromide.

Under the electric field, free negative ODNs moved to the positive electrode and displaced in the gel as a visual band (Figure 5, Lane A). As the proportion of MCH in the samples was increased, a decrease or absence of staining intensity of ODN as seen in lanes B to F was observed. This suggests that progressively increasing amount of ODN was retained by MCH in the wells as the proportion of MCH to ODN increased in the sample. As the *N*/*P* ratio reached 1 : 1 or above, ODN was completely complexed with MCH, as indicated by the lack of electrophoretic mobility; hence there is no free ODN available to move toward positive electrode leading to absences of visible ODN band in the gel. Thereafter at the charge ratio of 1 : 1 to 7 : 1, no band was visible indicating the enhanced efficiency of complexation (Lane C–F).

The electrophoretic mobility of ODN was retarded with increasing amount of MCH and retained at the top of the gel at ratio of 1 : 1 to 7 : 1. This suggests that MCH formed complexes completely with ODN at this ratio range. Although some amino groups are mannosylated leading to reduced charge density of MCH slightly, its ability to condense ODN was retained (Figure 5 lanes C–F). This characteristic is an essential requirement for condensing ODN and transfecting to the cells.

The article "Mannosylated Chitosan Nanoparticles for Delivery of Antisense Oligonucleotides for Macrophage Targeting" was retracted in 2021. Reasons: manipulated images; duplicated images; original data or images not available; concerns about the data.

### 7.2. Particle Size

Physicochemical properties of MCHODN nanoparticles with various charge ratios were characterized in terms of size and zeta potential (ZV). Literature reveals that the biological activities of the transfection reagents are highly associated with their physicochemical properties [112, 113].

Specific properties, such as particle size and surface charge of the complex, are necessary to assure its uptake by cells. In particular, the particle size of a complex is an important factor that influences the access and passage of the complex through the targeting site [103]. Mean particle diameter of MCHODN nanoparticles with different *N*/*P* ratios was determined by photon correlation spectroscopy (PCS) using Zetasizer as shown in Table 1.

It was observed that with increase in *N*/*P* ratio (from 1 : 1 to 7 : 1) that the mean particle size of MCHODN nanoparticles was decreased. It can be inferred that the particle size which was not more than 267 nm is indirectly proportional to the charge ratio (Table 1). When *N*/*P* ratio of MCHODN NPs was around 1, the nanoparticles size was above 250 nm. If the *N*/*P* ratio of MCH and ODN was increased from 1 to 7, the mean particle size was found to decrease from 267.12 ± 11.0 nm to 178.24 ± 7.4 nm. The possible reason could be that the polymer complexes with ODN through ionic interactions, and at higher *N*/*P* ratio, there are net electrostatic repulsive forces that can prevent aggregation among complexes. Similar trend was observed in the earlier report with galactosylated chitosan NPs carrying DNA [54].

Particle size can play an important role in influencing the transfection efficiency. The NPs with larger particle diameter bear disadvantage in the process of cell endocytosis, and, thus, the corresponding transfection efficiency may be poor [114, 115]. Further, with MCHODN NPs, the data represents suitable PI value for *N*/*P* ratio from 3 to 7 inferring to their homogenous nature.

### 7.3. Zeta Potential (ZV)

The zeta potential of the MCHODN NPs at various *N*/*P* ratios is given in Table 1. With increasing *N*/*P* ratio of MCH to ODN from 1 to 7, the zeta potential of the nanoparticles rapidly increased to positive values. It is inferred that the ZV is directly proportional to the charge ratio of nanoparticles. The increase in ZV was due to an increase in the positive charge density of the mannosylated chitosan. At charge ratio of 1 : 1 MCHODN NPs displayed negative ZV (−6.2 mV); however, with an increase in *N*/*P* ratio of MCH to ODN upto 7 : 1, NPs displayed positive zeta potential. Further, with increase in charge ratio from 3 : 1 to 7 : 1, the ZV raised from 8.9 mV to 14.5 mV. Complete shielding of negative charge of ODN was displayed in formulation with charge ratio 3 : 1. The results obtained are in accordance with the earlier reports [54, 62]. Upon self-assembly of ODNs and cationic polymer, the highly negative charge of ODNs gets neutralized rapidly, and the surface charge of the complex becomes positive at higher *N*/*P* ratio. A positive surface charge of polyplexes is necessary for binding to anionic cell surfaces, which consequently facilitates uptake by the cell [116, 117]. The surface charge of delivery systems carrying genetic material (DNA/ODNs) is one of the major factors influencing the biodistribution [118] and transfection efficiency [119]. Surface charge of polymer/ODN complexes plays an important role in the uptake of the complexes by cells and their physical stability in blood. Serum protein tends to adsorb strongly onto positively charged particles surfaces. This opsonization would lead to severe aggregation of the complexes and subsequent opsonization. It was reported that the slightly positive zeta potential resulted in the best transfection efficiency [120]; MCHODN NPs charge ratio above 1 is thought to be profitable for the ODN transfer into cells.

The article "Mannosylated Chitosan Nanoparticles for Delivery of Antisense Oligonucleotides for Macrophage Targeting" was retracted in 2021. Reasons: manipulated images; duplicated images; original data or images not available; concerns about the data.

These results also indicate that it is possible to formulate nanoparticles of a specific particle diameter by adjusting condensing conditions, such as the *N*/*P* ratio of the complexes, concentration of ODN, and concentration of MCH.

### 7.4. Shape and Surface Morphology

The formulated nanoparticles were morphologically examined by TEM at magnifications at 8000 (Figure 15(a)). TEM images reveal solid, consistent, and compact structure having a spherical shape. As depicted from earlier studies the formulations were in nanometric range. Nanoparticles had a dense and spherical shape which is in good agreement with the SEM photomicrograph (Figure 15(b)). Percent ODN association of selected MCHODN NP2 formulation was determined to evaluate the amount of ODN associated with MCH in nanoparticulate formulation. The optimum transfection efficiency of MCHODN NP formulations was achieved at charge ratio of MCH/ODN at 3 : 1. On the basis of transfection efficiency results, MCHODN NP2 formulation was opted for further* in vitro* and* in vivo* studies. The percent ODN association of MCH ODN NP2 was found to be 98.5. This suggests that almost all the ODN loads were condensed into NP.

### 7.5. Resistance of MCHNP/ODN against DNase I Digestion and Release Assay

The plasmid DNA is readily degraded by endonucleases such as DNase I [121], which is one of the obstacles for the delivery of gene* in vitro* or* in vivo*. Therefore, the stability in the presence of DNase I is one of the essential parameters of systemic gene delivery. The chitosan was used to condense plasmid DNA/ODN to protect them against DNase digestion [54, 67, 103, 122]. To investigate whether naked ODN as well as complexed ODN with mannosylated chitosan was stable against nuclease digestion, DNase I protection assay was carried out. The results indicated that naked ODN remained intact after DNase I treatment indicated by the presence of visual band in the gel and maintained its integrity (Figure 6(a), lane A) because phosphorothioate ODN is resistant to nuclease degradation.

The article "Mannosylated Chitosan Nanoparticles for Delivery of Antisense Oligonucleotides for Macrophage Targeting" was retracted in 2021. Reasons: manipulated images; duplicated images; original data or images not available; concerns about the data.

Figure 6(a), lanes A–F show that the free ODN, as well as ODN associated with MCHODN NPs at all *N*/*P* ratio, remained intact after treatment with DNase I enzyme and staining intensity in the well was increased on increasing the *N*/*P* ratio of MCH/ODN. Only single band was observed with free ODN in the gel, which reveals that the process of complexation with MCH does not affect the integrity of the ODN adversely rather it seems to offer protection. This suggests that ODN either in free form or in complexed form with mannosylated chitosan at various *N*/*P* ratios maintained their integrity and resistant to DNase I enzyme degradation.

In release assay, DNase I digested NPs suspension was treated with SDS to release ODN from complexes that was evaluated by agarose gel electrophoresis. The released ODN from nanoparticulate carriers displayed visual bands in the gel (Figure 6(b), lanes A–F). The results indicate that at 0.5 : 1 to 7 : 1 ratios of MCH/ODN, ODN remained intact after DNase and SDS treatment. This demonstrates that the process of complexation of mannosylated chitosan does not affect the ODN integrity adversely rather it seems to offer protection. Under the physiological conditions, where the nuclease concentration is markedly lower than the tested concentration, a formulation should render a significant protection to the ODNs. The results indicate that binding of ODNs to MCH was sufficient to provide protection against enzymatic degradation.

### 7.6. Stability of MCHODN NPs Formulation

#### 7.6.1. Dispersive Stability

The study was conducted with an objective to evaluate whether the formulations form self-aggregate or precipitate in phosphate buffer at room temperature. It is expected that the decrease in turbidity with duration of storage would indicate precipitate formation. From the present data (Figure 7) it can be inferred that the formulation MCHODN NP2 displayed steady values of absorbance till 1.5th day and thereafter slight decrease on 2nd day indicates precipitate formation. The results suggested that MCHODN NP2 formulation displayed appreciable stability during the study period.

The article "Mannosylated Chitosan Nanoparticles for Delivery of Antisense Oligonucleotides for Macrophage Targeting" was retracted in 2021. Reasons: manipulated images; duplicated images; original data or images not available; concerns about the data.

#### 7.6.2. Serum Stability

Stability of nanoparticles formulations MCHODN NP2 and free ODN were observed in presence of serum to investigate the behavior in physiological condition. Gel electrophoresis results revealed that up to 2nd day of incubation period at 37°C nanoparticles remained stable (Figure 8).

## 8. Cytotoxicity Assay

Cytotoxicity assay was conducted to evaluate the effect of polymer concentration on cell viability. MTT assay was performed to determine the cytotoxicity of MCH in two different cell lines, that is, Raw 264.7 cells and Hela cells, over a wide range of polymer concentration. MCH showed acceptable cell viability in both cell lines at lower concentration. MCH exhibited near about 88.4% cell viability at 200 *μ*g/mL in Raw 264.7 cells. The maximum cell viability 104.5% and 100.2% was observed at 10 *μ*g/mL with MCH in Raw 264.7 and Hela cells, respectively. It might be concluded that the cells growth is appreciable even at higher concentration of 200 *μ*g/mL with MCH (Figure 9). Chitosan is reported to bear low toxicity [67, 123] although few reports reveal a dose-dependent toxicity of chitosan at high doses* in vitro* [54]. In earlier reports, significantly higher cell viability of chitosan-treated cells was observed compared to PEI [98, 124]. In the present study, the cell viability further increased after mannosylation of chitosan. The cell viability of MCH (~85.0% of control) was significantly higher than that of CH (~60.2% of control) at a concentration of 100 *μ*g/mL in the Raw 264.7 cell lines; data not shown. As reported earlier, cationic polymers with high charge density have strong cell lytic and toxic properties and also a reduction of charge density resulted in reduced cell toxicity or increased cell viability [125]. Lower toxicity of MCH may be attributed to steric hindrance and the charge shielding effects offered by mannose moiety. Recent evidence suggests that the introduction of sugar into the polycations affects electrostatic interactions between anionic cell surfaces and cationic polymer. This leads to reduction of membrane damaging effects, which is a typical characteristic of polycationic molecules [126]. The results from present study are in accordance with the research work related to the polymeric nanoparticulate carriers for delivery of gene in earlier reports [62, 93, 127, 128]. The results further incept that modified chitosan being noncytotoxic, biocompatible, and safe vector might play a role of compatible gene delivery system. Therefore, nanosized MCHs are expected to be suitable carrier for gene therapy because of their favorable and acceptable physicochemical properties largely leading to their low cytotoxicity.

The article "Mannosylated Chitosan Nanoparticles for Delivery of Antisense Oligonucleotides for Macrophage Targeting" was retracted in 2021. Reasons: manipulated images; duplicated images; original data or images not available; concerns about the data.

To further evaluate the efficiency of mannosylated systems, the influence of various ODN concentrations associated with MCHODN NPs on the cell viability of Raw 264.7 macrophages cells was investigated using MTT assay.

The results are displayed in Figure 10. Raw 264.7 cells incubated with ODN formulations equivalent to 1 to 10 *μ*g ODN displayed variations. It was observed that more than 90% cells were viable at 1 *μ*g ODN concentration in case of MCHODN NPs. Sign of cytotoxicity was minimum in case of MCHODN NPs, when ODN concentration increased up to 10 *μ*g. More than 75% cells were viable at all the tested ODN concentrations with MCH.

Hashimoto et al. [95] studied the transfer of gene by DNA/mannosylated chitosan complexes into mouse peritoneal macrophages and it was reported that on increasing the DNA concentration from 1 to 10 *μ*g the cell viability of mannosylated chitosan/DNA complex was unchanged. It might be inferred that MCHODN NPs show significantly higher cell viability at all ODN concentrations (Figure 10). The cytotoxicity of pDNA/PEI complexes was reported to be higher [52, 123] as compared to that of pDNA/chitosan complexes [63, 129]. The mannosylation of chitosan further decreases the cytotoxicity and might significantly increase the transfection efficiency. The low cytotoxicity of MCHODN NPs might be due to its hydrophilic surface. It could be hypothesized that the hydrophilic surface of MCHODN NPs suppresses the formation of aggregation followed by nonspecific adhesion to the cell surface.

### 8.1. *In Vitro* Transfection Assay with Mannosylated Chitosan Nanoparticles

In order to evaluate the* in vitro* gene transfer capability of mannosylated chitosan nanoparticles, the transfection assay was carried out at different *N*/*P* ratio of MCH to ODN in Raw 264.7 cells and Hela cells.  Figure 11 suggests that transfection efficiency is dependent on charge ratio of MCH/ODN. There is significant increase in transfection efficiency of MCHODN NPs in Raw 264.7 cells from 28.78 ± 1.2 ng/10^6^ cells to 73.18 ± 4.2 ng/10^6^ cells on increasing *N*/*P* ratio of MCH and ODN from 1 : 1 to 3 : 1, whereas, on further increasing the *N*/*P* ratio to 5 : 1, a decrease in transfection efficiency to 63.08 ± 3.6 ng/10^6^ cells was observed and remained almost constant at ratio of 7 : 1. Maximum transfection efficiency was recorded at optimum *N*/*P* ratio of 3 : 1. Further, MCHODN NPs displayed approximately 3-fold higher transfection efficiency to that of free ODN.

The article "Mannosylated Chitosan Nanoparticles for Delivery of Antisense Oligonucleotides for Macrophage Targeting" was retracted in 2021. Reasons: manipulated images; duplicated images; original data or images not available; concerns about the data.

This might be due to the poor cellular uptake of ODN in free form because of its negative charge and hydrophilic nature [11]. The possible reason is that naked ODN gets degraded rapidly in presence of cellular enzymes unlike the one complexed to mannosylated chitosan [14]. It is expected that ODNs complexed to mannosylated chitosan get protective shielding against enzymatic degradation. The MCHODN NPs presents high density of mannose for interaction with cell surface. Raw 264.7 cells that express moderate mannose receptors might present higher opportunity for transfection of mannosylated system. Kim et al. [62] reported the utility of mannose receptor based endocytosis as they explored mannosylated chitosan nanoparticles for cytokine gene therapy. Also, in this context, Jiang et al. [127] explored mannosylated chitosan PEI grafts for DNA delivery exploiting mannose receptor. Few other applications of mannosylated cationic systems with enhanced transfection efficiency are reported [128, 130–132]. Macrophages and dendritic cells have substantial amount of mannose receptors on the surface, suggesting that MCH-mediated gene delivery may be induced by receptor-mediated endocytosis via surface-bound mannose receptors. The results substantiate the findings that mannosylated system is more effective for gene expression in Raw 264.7 cells than nonmannosylated systems.

The results from transfection assay at various *N*/*P* ratios using galactosylated chitosan for gene delivery are in accordance with the present results for mannosylated carriers [54, 67]. Literature cites that, for effective expression of gene, vehicle must protect the enzymatic degradation of gene [133]. The transfection efficiency of naked ODN, MCHODN NPs, and lipofectin/ODN complex in Raw 264.7 and Hela cells was also compared in order to demonstrate the effect of mannose on receptor mediated gene transfer. The differences in transfection efficiency in two cell lines are clearly observed as Raw 264.7 cell lines displayed significantly higher transfection at each *N*/*P* ratio as compared to Hela cells in which mannose receptors are not present (Figure 11).  Figure 12 demonstrates that transfection efficiency of MCHODN NP2 is much higher than naked ODN and similar to that of lipofectin. At optimum *N*/*P* ratio of 3 : 1, MCHODN NP2 displayed 2.53-fold higher transfection in Raw 264.7 cells than Hela cells. It indicates that the mannose ligand on MCHODN NPs played an important role in mannose receptors recognition and enhanced transfection in Raw 264.7 cell. There is no difference observed in case of MCHODN NPs and naked ODN in regard to transfection in Hela cells, which lacks mannose receptor on cell membrane surface. However, transfection efficiency of lipofectin/ODN complexes was found to be much higher as compared to MCHODN NPs. Kawakami and coworkers [72, 83] earlier emphasized that the mannose receptor-mediated pathway is more effective for gene expression in macrophages than the nonspecific pathway [134, 135]. These results suggest that the MCHODN NPs have the capability to transfect the cell lines with mannose selectively. Thus, MCHODN NPs are an efficient carrier for delivery of free ODN.

The article "Mannosylated Chitosan Nanoparticles for Delivery of Antisense Oligonucleotides for Macrophage Targeting" was retracted in 2021. Reasons: manipulated images; duplicated images; original data or images not available; concerns about the data.

#### 8.1.1. Competition Assay

For initial studies, Raw 264.7 macrophages cells expressing moderate mannose receptors were used and it was found that the enhanced cellular uptake of the MCHODN NPs is due to the mannose mediated endocytosis. The transfection activity of MCHODN NP2 prepared at a charge ratio of 3 : 1 was investigated in the presence of various amounts of mannose as a competitor for the nanoparticles and results are given in Figure 13 show the relationship between the transfection efficiency of ODN and MCHODN NP2 (*N*/*P* = 3) and the mannose inhibition concentration.

The transfection efficiency of MCHODN NP2 decreases when the concentration of mannose increases and transfection efficiency/uptake of MCHODN NP2 was inhibited about 50% at 20 mM concentration of mannose.

Our results clearly indicate that MCH-mediated ODN delivery was mannose receptor-dependent because mannose could block the binding in a concentration-dependent manner. In other words, the availability of mannose receptors is essential for entry of MCHODN NPs into macrophages through a receptor mediated delivery system. Our results are in accordance with the earlier reported work with mannosylated cationic polymer for DNA delivery [62, 93, 128, 136].

### 8.2. Cellular Uptake

Cellular uptake of FITC-ODN alone against MCHODN NPs was studied by fluorescent microscopy and confocal laser scanning microscopy following the incubation of Raw 264.7 cells with free ODN and nanoparticles formulations for 4 h at 37°C. Results shown in Figures 16(a) and 16(b) clearly exhibit an increased uptake of MCHODN NP2 compared to the FITC-ODN alone. Increased fluorescence in the cells displayed higher cell uptake of MCHODN NP2 as compared to free ODN as further confirmed by CLSM image (Figure 16(c)).

## 9. Antisense Activity

To investigate the inhibitory activity of ODN on LPS (lipopolysaccharide) stimulated TNF-*α* release, two different sequences of ODN, namely, TJU-2755 (complementary rat TNF-*α* mRNA) and TJU-2755-RD (Random), were used. In order to determine the potential inhibitory effect of oligonucleotides on LPS stimulated TNF-*α* release, free ODN and MCHODN NPs formulations were added to the cells simultaneously with LPS. Concentration of TNF-*α* after exposure to ODN either in free form or in NPs formulations measured using ELISA method displayed results as shown in Figure 14. The oligonucleotide (TJU-2755-ODN) was designed to target rat TNF-*α* mRNA. LPS was used to stimulate macrophage for secretion of cytokines, including TNF-*α*. Efficient delivery of ODN into macrophage is proposed to suppress the expression of TNF-*α* [137]. The concentration of TNF-*α* after LPS treatment was found to be 104.32 ± 7.6 ng/mL. As shown in the data, free ODN bear weak inhibitory effect on TNF-*α* expression, while MCH NPs could markedly promote ODN transfer into cells, which might block TNF-*α* gene expression. After exposure to various formulations, the TNF-*α* concentration was reduced to 92.42% and 43.96% (of control) with free ODN and MCHODNNP2, respectively. Transfection effect of MCH NPs as ODN carrier was higher than free ODN.

The article "Mannosylated Chitosan Nanoparticles for Delivery of Antisense Oligonucleotides for Macrophage Targeting" was retracted in 2021. Reasons: manipulated images; duplicated images; original data or images not available; concerns about the data.

To evaluate the inhibitory effect of TJU 2755 ODN on rat TNF-*α* production, a control random scrambled sequence of TJU 2755 was used with MCH NPs formulation. Results shown in Figure 14 indicate that MCHODN NP2 containing TJU 2755 ODN (complementary sequences of rat TNF-*α* mRNA) displayed significant reduction (approx. 55% of control) in rat TNF-*α* production induced by LPS, whereas MCHODN NP2 containing TJU2755 RD sequence showed no inhibitory effects on TNF-*α* production. The results suggest that suppression of TNF-*α* production is dependent on the ODN sequence.

## 10. Conclusion

In the present work, mannosylated low molecular water soluble chitosan was successfully prepared and found as a suitable targeting gene delivery carrier to macrophages. It displayed good capacity to form nanoconstructs with oligonucleotide and showed suitable physiochemical properties for gene delivery system. These mannosylated nanoconstructs had no cytotoxicity and exhibit much higher gene transfer efficiency on Raw 264.7 cells. TJU 2755 antisense oligonucleotide displayed antisense activity by reducing the LPS induced serum TNF-*α* in 264.7 cells. Mannosylated chitosan displays potential regarding safe and efficient gene targeting to the macrophages.

## Figures and Tables

**Figure 1:** FTIR spectrum of chitosan.

**Figure 2:** ^1^H NMR spectrum of chitosan.

**Scheme 1:** Reaction scheme for MCH Preparation.

**Figure 3:** FTIR spectrum of mannosylated chitosan.

**Figure 4:** ^1^H NMR spectrum of mannosylated chitosan.

**Figure 5:** Gel retardation assay of MCHODN NPs; lane A: free ODN; lanes B–F: MCHODN NPs at *N*/*P* ratio of 0.5 : 1, 1 : 1, 3 : 1, 5 : 1, and 7 : 1.

The article "Mannosylated Chitosan Nanoparticles for Delivery of Antisense Oligonucleotides for Macrophage Targeting" was retracted in 2021. Reasons: manipulated images; duplicated images; original data or images not available; concerns about the data.

**Figure 6:** (a) MCHODN NPs that were separately incubated with DNase I. (b) 1.0% SDS was added to DNase I treated samples in the MCHODN NPs. Lane A: free ODN; lanes B–F: MCHODN NPs with increasing ratio (0.5, 1, 3, 5, and 7).

**Figure 7:** Stability of MCHODN NP2 formulations in 10 mM phosphate buffer containing 150 mM NaCl.

**Figure 8:** Gel electrophoresis of MCHODN NP2 after incubation at 37°C under mild agitation with increase storage period. Lane A: nanoparticles prepared immediately prior to gel analysis (initial); lanes B–E: nanoparticles with increasing incubation period (0.5, 1, 1.5, and 2 days); lane F: free ODN.

**Figure 9:** Cell Viability studies of MCH at different polymer concentration in Raw 264.7 and Hela cells (*n* = 3).

**Figure 10:** Cell viability study of MCHODN NPs with different ODN concentration in Raw 264.7 cells after 24 h (*n* = 3).

**Figure 11:** Transfection efficiency of MCHODN nanoparticles at different *N*/*P* ratio in Raw 264.7 cells and Hela Cells (*n* = 3).

**Figure 12:** Comparative study of transfection efficiency in Raw 264.7 cells and Hela cells with free ODN and MCHODN NP2 and at *N*/*P* ratio of 3 : 1 (*n* = 3). Transfection efficiency using Lipofectin 2000 was set as a positive control.

**Figure 13:** Competition assay of MCHODN NP2 (*N*/*P* = 3) in Raw 264.7 cells with different concentration of mannose.

**Figure 14:** TNF-*α* expression profile of transfected Raw 264.7 cells with free ODN and MCHODN NP2 after stimulation of cells with 100 ng/mL LPS (*n* = 3), ^#^ *Control cells treated with PBS* +* LP.*

**Figure 15:** (a) TEM photomicrograph magnification (×80000), (b) SEM photomicrograph of MCHODN NP2.

**Figure 16:** Fluorescent microscopic images of Raw 264.7 cells treated with (a) Free ODN and (b) MCHODN NP2. (c) Confocal laser scanning microscopic image of Raw 264.7 cells treated with MCHODN NP2.

**Table 1:** The composition and characterization of MCHODN NPs (*n* = 3).

Formulation codes	*N*/*P* ratio of MCH to ODN	Particle size (nm)	Zeta potential (mV)	Polydispersity index (PI)
MCHODN NP1	1 : 1	267.12 ± 11.0	−6.2 ± 0.02	0.38
MCHODN NP2	3 : 1	192.48 ± 4.8	+8.9 ± 0.82	0.12
MCHODN NP3	5 : 1	187.16 ± 5.6	+12.6 ± 0.64	0.16
MCHODN NP4	7 : 1	178.24 ± 7.4	+14.2 ± 0.46	0.20

Values expressed as Mean ± SD.
